# UCH-L1 Inhibitor Alleviates Nerve Damage Caused by Moyamoya Disease

**DOI:** 10.1155/2024/2550642

**Published:** 2024-07-25

**Authors:** Minghua Xu, Xiaomin Zhao, Jiang Zhao, Zhisheng Tan, Chengshi Zhang, Yun Huang, Huiping Zhong, Meifeng Guo, Chen Zhang, Ping Ye, Wentao Zheng

**Affiliations:** ^1^ Intensive-Care Unit Punan Branch of Renji Hospital Shanghai Jiao Tong University School of Medicine, Shanghai 200125, China; ^2^ Department of Neurosurgery Punan Branch of Renji Hospital Shanghai Jiao Tong University School of Medicine, Shanghai 200125, China; ^3^ Geriatric Department 920th Hospital of Joint Logistics Support Force, PLA, Kunming 650200, Yunnan, China; ^4^ Department of Respiratory Punan Branch of Renji Hospital Shanghai Jiao Tong University School of Medicine, Shanghai 200125, China; ^5^ Department of Clinical Laboratory Punan Branch of Renji Hospital Shanghai Jiao Tong University School of Medicine, Shanghai 200125, China

## Abstract

**Background:**

Moyamoya disease (MMD) leads to nerve injury. Exosomes are touted as bio-shuttles for the delivery of distinct biomolecules inside the cells. Recently, UCH-L1 was shown to play a vital role in nerve injury. However, it is still unknown whether UCH-L1 can improve the nerve injury of MMD.

**Materials and Methods:**

Exosomes were isolated from the serum of patients with MMD and healthy controls. The total RNA was extracted from the exosomes, and the level of GFAP and UCH-L1 between the serum exosomes of the two groups was analyzed by a quantitative reverse transcription-polymerase chain reaction and western blot. Exosome labeling and uptake by SH-SY5Y cells were observed by confocal laser microscopy. Cell counting kit-8 assay and flow cytometry were used to determine the viability and apoptosis of SH-SY5Y cells, respectively.

**Results:**

Exosomes were successfully isolated and identified from serum. The expression of GFAP and UCH-L1 was significantly higher in the serum-derived exosomes from MMD patients compared with the healthy controls (*P*  < 0.05). Compared to the blank and control exosome group, serum-derived exosomes from MMD significantly suppress cellular vitality and promote apoptosis of SH-SY5Y cells, while the use of LDN-91946, a specific inhibitor of UCH-L1, could reverse the effects induced by serum-derived exosomes from MMD.

**Conclusion:**

UCH-L1 inhibitor could reverse MMD-induced inhibition of SH-SY5Y cell viability and promotion of apoptosis. UCH-L1 may be a therapeutic target for the treatment of nerve damage caused by MMD.

## 1. Introduction

Moyamoya disease (MMD) is a progressive cerebrovascular disorder characterized by bilateral steno-occlusive changes at the terminal portion of the internal carotid artery and an anomalous vascular network at the base of the brain [1, 2]. Its prevalence is highest in East Asian nations, with an annual incidence of 0.43 per 100,000 in China and 0.54 per 100,000 in Japan, surpassing significantly that in the United States (0.086 per 100,000) and Europe (0.3 per 100,000) [3, 4, 5, 6]. Currently, surgical intervention serves as the primary treatment approach for MMD, encompassing indirect revascularization, direct revascularization, and combined revascularization [7, 8]. While surgical treatments have demonstrated definite efficacy, a consensus on the optimal surgical approach remains elusive [9, 10]. Moreover, various complications may arise following vascular reconstruction, including cerebral infarction, transient ischemic attack, intracerebral hemorrhage, hyperperfusion syndrome, impaired wound healing, and subdural effusion [11, 12]. Diagnosis of postoperative complications in patients with MMD primarily relies on cranial CT scans, ultrasound examinations, magnetic resonance imaging, and angiography [13, 14]. Due to the incomplete understanding of the specific pathogenesis of MMD and the rapid progression of various brain impairments after surgery, symptoms typically reach their peak within seconds [15, 16]. Therefore, early prediction of the degree of nerve injury in MMD patients can help to better guide clinical treatment and improve patient prognosis.

Recent clinical trials have delved into the dependability and precision of diverse brain-specific biomarkers as indicators of the progression and prognosis of brain and nerve injuries [17, 18, 19]. As the promising candidate biomarkers, UCH-L1 and GFAP, in conjunction, have recently garnered approval from the US Food and Drug Administration (FDA) for the evaluation of intracranial injury in patients with traumatic brain injury [20]. GFAP, an astrocyte-type III intermediate filament protein with specificity for brain tissue, is regarded as a distinctive marker of activated astrocytes [21]. GFAP serves to uphold the cytoskeletal structure of glial cells and fortify their mechanical strength [22]. UCH-L1, belonging to the UCH family of ubiquitination enzymes in the ubiquitin-proteasome system, exhibits abundant expression in the brain, constituting approximately 5% of the total protein content in the brain [23, 24]. UCH-L1 assumes a vital role in upholding neuronal integrity and viability [25]. Myriad experimental and clinical investigations have demonstrated elevated levels of GFAP and UCH-L1 in cerebrospinal fluid (CSF) and blood samples from individuals following traumatic brain injury and stroke, with notable correlations established between these biomarkers and the severity and outcome of the respective conditions [26, 27]. Furthermore, GFAP and UCH-L1 have exhibited remarkable accuracy in predicting unfavorable neurological outcomes [28].

In recent times, exosomes have garnered considerable attention within the scientific realm due to their burgeoning involvement in intercellular communication, encompassing a wide array of physiological and pathological processes spanning the entirety of the organism [29]. Notably, exosomes have been implicated in various neurodegenerative disorders, including Parkinson's, prion diseases, and Alzheimer's disease, wherein they have been observed to harbor aggregated forms of alpha-synuclein, Prion protein, Amyloid precursor protein, and phosphorylated tau, respectively [30, 31]. In this study, we extracted exosomes from the serum of MMD patients and healthy controls and examined the expression of GFAP and UCH-L1 in exosomes. The exosomes were then cocultured with SH-SY5Y cells, and the biological functions of serum-derived exosomes from MMD patients on SH-SY5Y cells were analyzed.

## 2. Materials and Methods

### 2.1. Study Subjects

Blood samples were collected from a total of 18 MMD patients and 18 healthy controls. The inclusion criteria encompassed the following: (1) digital subtraction angiography confirming the presence of MMD and patients meeting the Guidelines for Diagnosis and Treatment of Moyamoya Disease (Spontaneous Occlusion of the Circle of Willis); (2) patients within the age range of 30–70 years. MMD is a cerebrovascular disorder of unknown etiology. For accurate diagnosis, it is imperative to exclude conditions that manifest with similar vascular anomalies, including atherosclerosis, autoimmune diseases, meningitis, brain neoplasms, Down's syndrome, neurofibromatosis type 1 (von Recklinghausen's disease), sickle cell disease, traumatic brain injury, and cerebrovascular lesions post cranial irradiation. Additionally, individuals receiving long-term oral immunosuppressive therapy, those prescribed antiplatelet or anticoagulant medications, and patients undergoing chronic dialysis treatment were also excluded to mitigate the influence of these confounding factors on the secretion and content of exosomes. The control and MMD groups were matched in terms of age, sex, and body mass index. The foundational features of the MMD group and the control group are documented in Table 1. All experiments performed were approved by the Ethics Committee of the Punan Branch of Renji Hospital, Shanghai Jiao Tong University School of Medicine. All patients and healthy volunteers provided informed consent. Peripheral blood samples were collected in green-top vacutainer tubes. Specimens were centrifuged at 2,000 × *g* for 15 min, and the plasma was removed and aliquoted for storage at −80°C until further use.

### 2.2. Cell Culture and Cell Treatment

The SH-SY5Y cells were acquired from FuHeng Biology (Shanghai, China). Cells were cultured in Dulbecco's modified Eagle's medium supplemented with 10% fetal bovine serum (Gibco, Grand Island, NY, USA) and 1% penicillin/streptomycin (Gibco, Grand Island, NY, USA) at 37°C with 5% CO_2_.

For the cell treatment, 4 × 10^4^ SH-SY5Y cells were seeded into 24-well plates and placed in a cell incubator for an overnight period of static incubation. About 20*μ*g/mL exosomes or LDN-91946 were added to the culture medium. The cells were collected for subsequent experiments after incubation for 48 hr.

### 2.3. Isolation of Exosomes

The serum samples were thawed on a bed of ice. Next, the serum was subjected to centrifugation at 500× *g* for 10 min, and the supernatant was obtained. Following this, a sequence of low-speed centrifugation steps (2,000× *g* for 30 min, 10,000× *g* for 30 min) was performed to remove cellular debris. The resulting supernatant was then passed through a 0.22 *μ*m membrane filter (Jet Biofil, Guangzhou, China) for filtration. The filtrate was subsequently subjected to ultracentrifugation at 120,000× *g* for 70 min. The resulting supernatant was aspirated and discarded to obtain exosome pellets. Nanoparticle tracking analysis (NTA) and transmission electron microscopy (TEM) were used to identify exosomes.

### 2.4. Exosomes Uptake Assay

Exosome uptake of SH-SY5Y cells was analyzed by PKH67 staining assay using the kit (PKH67GL-1KT; Sigma–Aldrich, United States) according to the manufacturer's instructions. Briefly, Diluent C (400 *μ*L) was added to the exosomes (100 *μ*L), and then 500 *μ*L of Diluent C and 2 *μ*L PKH67 dye were added. The mixture was incubated at room temperature for 5 min. Subsequently, 1% bovine serum albumin (l mL BSA; Sigma–Aldrich, United States) was added to bind excess dye. The mixture was centrifuged at 120,000× *g* for 60 min to remove the supernatant, and the sediment (PKH67-labeled exosomes) was resuspended in PBS for use.

The SH-SY5Y cells were seeded into 24-well plates and cultured overnight in a serum-free medium. The next day, PKH67-labelled exosomes were added to each well and cocultured with SH-SY5Y cells for 24 hr. After washing three times with PBS, the SH-SY5Y cells were fixed in 4% paraformaldehyde for 20 min. After washing, the cells were stained with 4, 6-diamidino-2-phenylindole (Vector Labs, CA, USA) and observed under a laser scanning confocal microscope (TCS SP8, Leica Microsystems, Inc., United States).

### 2.5. Western Blot

Exosomes were lysed in RIPA Buffer (P0013B, Beyotime, China). Protein concentrations were determined utilizing a BCA Protein Assay Kit (G2026, Servicebio, China). Sodium dodecyl sulfate-polyacrylamide gel electrophoresis was employed for protein separation, followed by transfer onto polyvinylidene difluoride membranes. The membranes were subsequently immersed in 5% skim milk for 1 hr to block nonspecific binding. Afterward, the membranes were incubated overnight at 4°C with primary antibodies (anti-CD9 (1 : 1,000; Proteintech, 20597-1-AP), anti-HSP70 (1 : 2,000; Proteintech, 10995-1-AP), anti-TSG101 (1 : 1,000; Proteintech, 28283-1-AP), anti-GAPDH (1 : 50,000; Proteintech, 60004-1-Ig), anti-GFAP (1 : 2,000; Proteintech, 16825-1-AP), and anti-UCH-L1 (1 : 3,000; Proteintech, 14730-1-AP)). Subsequently, the membranes were incubated at 37°C for 1 hr with horseradish peroxidase-conjugated secondary antibodies (anti-rabbit IgG, 111-035-003, or anti-mouse IgG, 115-035-003, Jackson ImmunoResearch, 1 : 5,000). Visualization of the protein bands was accomplished using an enhanced chemiluminescence kit (Beyotime, China), and the grayscale density of the bands was quantified utilizing ImageJ software.

### 2.6. Reverse Transcription-Quantitative Polymerase Chain Reaction (RT-qPCR)

Total RNA was extracted using Trizol Reagent (Invitrogen). The extracted total RNA was then subjected to reverse transcription utilizing the PrimeScript RT Reagent Kit (Takara, Japan) according to specific protocols. Subsequently, RT-qPCR was performed employing the SYBR Green PCR Kit (Thermo Fisher Scientific, USA). The relative standard curve method (2^−*ΔΔ*CT^) was employed to ascertain the relative mRNA expression, with GAPDH serving as the reference gene. Detailed primer sequences are shown in Table 2.

### 2.7. CCK-8 Assay

The cell viability was assessed utilizing the Cell Counting Kit-8 (CCK-8, Beyotime Biotechnology, Shanghai, China) according to the guidelines provided by the manufacturer. Briefly, the cells were inoculated at a density of 1 × 10^4^ per well in 96-well plates overnight. Subsequently, the cells were treated with different treatments for 48 hr, followed by the addition of 10 *μ*L of CCK-8 reagent. After incubation for 2 hr, the absorbance at 450 nm was measured using a microplate reader (Multiskan MK3; Thermo Fisher Scientific).

### 2.8. Flow Cytometry

To evaluate cell apoptosis in the SH-SY5Y cells subjected to different treatments, the Annexin V-FITC/PI apoptosis assay kit (Beyotime Biotechnology) was employed, following the manufacturer's instructions. The cells were collected and centrifuged at 1,000× *g* for 5 min. After PBS washing, the cells were suspended in 1x binding buffer (195 *μ*L). Subsequently, 5 *μ*L of FITC-Annexin V and 5 *μ*L of PI (50 *μ*g/mL) were added to the cell suspension. The cells were then incubated for 15 min at 25°C in a dark environment. Finally, the cells were analyzed using a flow cytometer (FACSCalibur, BD Biosciences).

### 2.9. Statistical Analysis

The data were analyzed using GraphPad Prism 8.0 software and presented as the mean ± standard deviation. Differences between two groups were assessed using *t*-tests, while a one-way analysis of variance was utilized to identify differences among three or more groups. Statistical significance was defined as *P* < 0.05.

## 3. Results

### 3.1. Identification of Serum-Derived Exosomes

Serum-derived exosomes were analyzed and verified by TEM, NTA, and western blot. The presence of exosomes was affirmed by the discerning eye of TEM, which revealed the presence of cup-shaped bilayer vesicles (Figure 1(a)). The exosomal surface markers CD9, HSP70, and TSG101 can be found in exosomes through western blot (Figure 1(b)). The NTA results showed that the average diameters of exosomes were 132.3 and 143.5 nm in the MMD and control groups, respectively (Figure 1(c)). All these data indicate that exosomes were successfully isolated.

### 3.2. Expression of Brain Injury Markers in Serum-Derived Exosomes from Patients with MMD

To further explore the expression of the brain-specific biomarkers in the patients with MMD, we detected the expression of UCH-L1 and GFAP by RT-PCR. Both the RT-PCR and western blot analyses demonstrated a significant upregulation of GFAP and UCH-L1 expression in the serum-derived exosomes from MMD patients compared to the control counterpart (*P* < 0.05, Figure 2).

### 3.3. Cellular Uptake of Exosomes

In order to confirm whether exosomes could be taken up by SH-SY5Y cells, PKH26 was utilized to label the exosomes, which were subsequently cocultured with the SH-SY5Y cells. Laser scanning confocal microscopy demonstrated that labeled exosomes were taken up by SH-SY5Y cells (Figure 3).

### 3.4. LDN-91946 Reverses the Effects of Serum-Derived Exosomes from MMD Patients on SH-SY5Y Cell Proliferation and Apoptosis

Subsequently, the biological functions of serum-derived exosomes from MMD patients on SH-SY5Y cells were investigated. The CCK-8 revealed that serum-derived exosomes from MMD patients significantly suppressed cellular vitality when compared to the blank and control exosome groups (*P* < 0.05, Figure 4). However, the addition of LDN-91946 (a specific inhibitor of UCH-L1) reversed the diminished cellular vitality caused by serum-derived exosomes from MMD patients. Furthermore, flow cytometry analysis demonstrated that serum-derived exosomes from MMD patients substantially increased the level of cellular apoptosis in comparison to the blank and control exosome groups (*P* < 0.05, Figure 5). Nevertheless, the introduction of LDN-91946 countered the escalated cellular apoptosis induced by serum-derived exosomes from MMD patients. These findings indicate that LDN-91946 possesses the ability to counteract the impact of serum-derived exosomes from MMD patients on the proliferation and apoptosis of SH-SY5Y cells.

## 4. Discussion

MMD is a cerebrovascular disorder characterized by progressive stenosis or occlusion of the internal carotid artery and/or its terminal branches, leading to an aberrant development of compensatory vascular networks comprising delicate cerebral vessels known as “moyamoya vessels” at the base of the brain [1]. Revascularization stands as the most efficacious approach to restore blood supply and enhance cerebral perfusion, thereby preventing secondary strokes in ischemic MMD and stabilizing cerebrovascular hemodynamics to regress delicate moyamoya vessels and avert hemorrhagic events [32, 33]. Despite surgical revascularization being the most successful modality in augmenting cerebral perfusion and diminishing the incidence of stroke in MMD patients, the occurrence of complications such as hyperperfusion syndrome, cerebral infarction, and epilepsy remains high due to hemodynamic irregularities [34]. Hence, the early prognostication of the extent of neural injury in patients holds paramount importance in guiding clinical interventions and improving patient prognosis. In this study, we successfully extracted exosomes from the serum of MMD patients and healthy controls. Notably, the expression levels of GFAP and UCH-L1 in serum-derived exosomes from MMD patients were significantly elevated compared to those in the control group. Furthermore, we discovered that inhibition of UCH-L1 (LDN-91946) reversed the impact of serum-derived exosomes from MMD patients on the proliferation and apoptosis of SH-SY5Y cells.

Exosomes have emerged as crucial mediators of intercellular communication within the nervous system, facilitating interactions between neurons, astrocytes, and neurovascular endothelial cells [35]. Exosomes hold immense promise as a source of biomarkers for the early detection and management of various pathological conditions, including cancer, neurodegenerative disorders, and infections [36]. Exosomes can be isolated from various body fluids, such as serum, urine, CSF, semen, saliva, amniotic fluid, and bile [37]. The gold standard method for exosome isolation involves a series of ultracentrifugation steps or separation using a sucrose density gradient centrifugation technique [38]. Subsequently, the characterization of exosomes is typically performed using electron microscopy and particle sizing analysis. Besides, different marker proteins can be used to identify exosomes depending on their source of isolation, and some common markers include tetraspanins, Alix, p63, CD63, CD9, CD81, and Hsp70 [39]. In our study, we employed ultracentrifugation to isolate exosomes and confirmed the successful isolation of exosomes from serum using TEM, NTA, and western blot.

Studies have revealed a correlation between neurological biomarkers, namely GFAP and UCH-L1, and the manifestation of neurological symptoms [40]. Both UCH-L1 and GFAP levels have been found to be associated with brain injury [20]. UCH-L1, a neuron-specific cytoplasmic enzyme abundantly present in neurons, has exhibited heightened concentrations in CSF and blood, which have been linked to neuronal degradation and increased permeability of the blood–brain barrier [41]. Various neurological disorders, including aneurysmal subarachnoid hemorrhage, traumatic brain injury, stroke, and neonatal hypoxic-ischemic encephalopathy, have shown elevated UCH-L1 concentrations [42, 43]. Moreover, research has indicated that the decline in UCH-L1 activity leads to multiple dysfunctions, such as oxidative stress and neuronal injury, primarily resulting from misfolded or damaged proteins [24, 44]. Consequently, these dysfunctions are likely propelled by intracellular aggregates, such as Lewy bodies in the case of *α*-synuclein, leading to neurodegeneration and, ultimately, cell death [45]. GFAP, on the other hand, is a structural protein found in astrocytes, which is released at higher levels during brain injury and degeneration [46]. In the early stages of brain injury, astrocytes play a crucial role in safeguarding brain tissue, and the expression level of GFAP partially reflects the extent of damage to brain nerve function [47]. However, as the ailment progresses, the formation of glial scars hinders nerve synapse regeneration and impedes nerve repair. The expression level of GFAP, to some extent, reflects the brain's plasticity for nerve repair [48]. Studies have demonstrated that in cases of central nervous system damage or ailment, GFAP enters the injured brain tissue, making its way into the CSF and blood, resulting in varying degrees of GFAP presence in the CSF and blood [49]. Consistent with previous research findings, this study discovered a significant upregulation of GFAP and UCH-L1 expression in serum-derived exosomes from MMD patients compared to the control group.

Moreover, the results shed new light on the role of serum-derived exosomes from MMD patients in affecting the cellular vitality and apoptosis levels of SH-SY5Y cells. Our findings reveal that serum-derived exosomes from MMD significantly suppress cellular vitality and promote apoptosis of SH-SY5Y cells, suggesting that MMD causes neurological damage. Interestingly, we found that the use of LDN-91946, a specific inhibitor of UCH-L1, could reverse the effects induced by these exosomes. The UCH-L1 enzyme is known for its role in protein degradation and has been implicated in various pathological conditions, including neurodegenerative diseases [45]. The ability of LDN-91946 to counteract the impact of MMD patient-derived exosomes implies that UCH-L1 might be involved in the mechanism underlying these effects. This raises the possibility that UCH-L1 could be a potential therapeutic strategy for nerve injury in MMD patients.

Despite these promising findings, it is important to acknowledge the limitations of our study. The in vitro nature of our experiments means that further research, particularly in vivo studies and clinical trials, is required to validate our findings and fully elucidate the role of exosomes and UCH-L1 in MMD. Moreover, it would be beneficial to further explore the contents of these exosomes to identify the specific molecules responsible for their effects on SH-SY5Y cells.

## 5. Conclusions

In conclusion, our findings revealed that serum-derived exosomes from MMD patients can induce elevated expression of GFAP and UCH-L1, leading to significant inhibition of cellular viability and promotion of apoptosis in SH-SY5Y cells. However, the utilization of a UCH-L1-specific inhibitor, LDN-91946, can reverse these exosome-induced effects. Our discoveries suggest a potential therapeutic role for UCH-L1 inhibitors in alleviating neurodegeneration caused by MMD. This unveils novel opportunities for the development of targeted therapies in MMD. Nonetheless, further research is imperative to validate these findings and elucidate the precise underlying mechanisms involved.

## Figures and Tables

**Figure 1:** Plasma-derived exosomes were identified: (a) transmission electron microscopy image of exosomes isolated from plasma; (b) the size distribution of exosomes determined by nanoparticle tracking analysis; (c) the images of exosome-specific CD9, HSP70, and TSG101 proteins examined by western blot.

**Figure 2:** RT-qPCR (a) and western blot (b) were performed to analyze the expression of UCH-L1 and GFAP.  ^*∗*^*P* < 0.05, compared with control-exosomes group.

**Figure 3:** Plasma-derived exosomes were stained by PKH67 to assess the cellular uptake of SH-SY5Y cells.

**Figure 4:** Cell viability was detected using CCK-8 assay.  ^*∗*^*P* < 0.05, compared with blank group. ^#^*P* < 0.05, compared with control-exosomes group. ^&^*P* < 0.05, compared with MMD-exosomes group.

**Figure 5:** Cell apoptosis was detected using flow cytometry.  ^*∗*^*P* < 0.05, compared with blank group. ^#^*P* < 0.05, compared with control-exosomes group. ^&^*P* < 0.05, compared with MMD-exosomes group.

**Table 1:** Clinical features of patients with moyamoya disease and control group.

Clinical features	MMD (*N* = 18)	Control group (*N* = 18)	*P*-value
Mean age (years)	44.72 ± 11.52	38.67 ± 6.64	0.067
Female sex	13 (72.22%)	12 (66.67%)	0.717
BMI	21.58 ± 1.03	22.16 ± 1.04	0.1

**Table 2:** Primer sequences in the study.

Gene	Forward primer and reverse primer (5′–3′)
GFAP-hF	AGGTCCATGTGGAGCTTGAC
GFAP-hR	GCCATTGCCTCATACTGCGT
UCH-L1-hF	CCTGTGGCACAATCGGACTTA
UCH-L1-hR	CATCTACCCGACATTGGCCTT
GAPDH-hF	TGACAACTTTGGTATCGTGGAAGG
GAPDH-hR	AGGCAGGGATGATGTTCTGGAGAG

## Data Availability

The datasets generated and/or analyzed during the current study are available from the corresponding author upon reasonable request.
